# ECG-Based Multiclass Arrhythmia Classification Using Beat-Level Fusion Network

**DOI:** 10.1155/2023/1755121

**Published:** 2023-11-29

**Authors:** Junyuan Jing, Jing Zhang, Aiping Liu, Min Gao, Ruobing Qian, Xun Chen

**Affiliations:** ^1^School of Information Science and Technology, University of Science and Technology of China, Hefei 230027, China; ^2^Department of Electrocardiogram, The First Affiliated Hospital of USTC, Division of Life Sciences and Medicine, University of Science and Technology of China, Hefei 230001, Anhui, China; ^3^Department of Neurosurgery, The First Affiliated Hospital of USTC, Division of Life Sciences and Medicine, University of Science and Technology of China, Hefei 230001, Anhui, China

## Abstract

Cardiovascular disease (CVD) is one of the most severe diseases threatening human life. Electrocardiogram (ECG) is an effective way to detect CVD. In recent years, many methods have been proposed to detect arrhythmia using 12-lead ECG. In particular, deep learning methods have been proven to be effective and have been widely used. The attention mechanism has attracted extensive attention in many fields in a series of deep learning methods. Off-the-shelf solutions based on deep learning and attention mechanism for ECG classification mostly give weights to time points. None of the existing methods were considered using the attention mechanism dealing with ECG signals at the level of heartbeats. In this paper, we propose a beat-level fusion net (BLF-Net) for multiclass arrhythmia classification by assigning weights at the heartbeat level, according to the contribution of the heartbeat to diagnostic results. This algorithm consists of three steps: (1) segmenting the long ECG signal into short beats; (2) using a neural network to extract features from heartbeats; and (3) assigning weights to features extracted from heartbeats using an attention mechanism. We test our algorithm on the PTB-XL database and have superiority over state-of-the-art performance on six classification tasks. Besides, the principle of this architecture is clarified by visualizing the weight of the attention mechanism. The proposed BLF-Net is shown to be useful and automatically provides an effective network structure for arrhythmia classification, which is capable of aiding cardiologists in arrhythmia diagnosis.

## 1. Introduction

Cardiovascular disease (CVD) is at high risk of leading to death. According to the World Health Organization (WHO), in 2019, an estimated 17.9 million individuals died from CVDs, representing 32% of global deaths [1]. In particular, sudden cardiac deaths account for roughly 50% of all fatalities due to cardiovascular disease, with cardiac arrhythmias accounting for about 80% of them [2]. Electrocardiogram (ECG) is widely used for recording the heart's electrical activities, which can reflect the physical condition of humans. ECG is noninvasive and inexpensive. It is obtained by electrodes attached to the skin. The standard ECG has 12 leads, namely, I, II, III, avR, avL, avF, V1, V2, V3, V4, V5, and V6. Automatic arrhythmia detection using ECG has become increasingly important. It can assist doctors in treating patients and provide helpful information about heart conditions for ordinary people with wearable devices.

ECG signal has its periodicity due to the regular electrical activity of the heart. A typical ECG signal record is composed of several heartbeats. These heartbeats are closely related physiologically and temporally. On the one hand, each beat of the ECG signal can be divided into PRQST waves according to different physiological meanings. Depolarization of the right atrium is responsible for the first half of the P wave, while depolarization of the left atrium is responsible for the second half. Depolarization of the middle of the left side of the interventricular septum causes the QRS complex's initial 0.01 second. Depolarization of the endocardium of both ventricles produces the next few milliseconds of the QRS complex. Depolarization of a smaller portion of the right ventricle and a larger portion of the left ventricle follows. The final few milliseconds of the QRS complex are caused by depolarization of the basilar region of the left ventricle. The T wave is created by the ventricles repolarizing [3].

In the past few decades, a large number of arrhythmia classification methods have been proposed. Technically, a typical method includes preprocessing, feature extraction, and feature classification. Feature extraction is the most sophisticated step because we need to choose a set of features manually. Therefore, ECG classification based on deep neural networks (DNNs), which have the capability of automatic feature extraction, has attracted much attention and many DNN-based arrhythmia classification works have been proposed.

Since each beat has the same structure, a novel method using the beat-level attention fusion network for multiclass arrhythmia classification is proposed by exploiting this feature. Our method can be divided into three steps: (1) segmentation, (2) beat-level feature extraction, and (3) interbeat feature fusion. The segmentation module transforms ECG signals into different heartbeats. Beat-level feature extraction module extracts features from heartbeats. Interbeat feature fusion module fuses beat-level features into global features that incorporate information about the whole ECG signal by considering the contribution of the heartbeat to diagnostic results. The main contributions of our algorithm are stated as follows. The model BLF-Net is proposed by utilizing the attention mechanism at the level of heartbeat instead of the time point. The attention mechanism gives weights for different beats in an ECG signal. The purpose is to focus on the informative beats and suppress less useful beats among one ECG signal. This model outperforms the state-of-the-art models in terms of arrhythmia detection. Besides, this model provides a new perspective for arrhythmia detection. That is, an ECG signal can be dealt with the level of heartbeats and attention can be utilized to fuse features extracted from each beat.

## 2. Related Works

Traditional methods are required to extract features manually. Typical features extracted manually are statistical features [4], morphological features [5, 6], P-QRS-T features [7, 8], and wavelet features [9, 10]. Also, dimensionality reduction methods can be exploited for extracting useful information, such as principal component analysis (PCA) [11], independent component analysis (ICA) [12, 13], and linear discriminant analysis (LDA) [14, 15]. After extracting features, there are varieties of classifiers to be chosen from. Commonly used techniques are support vector machine (SVM) [16, 17], artificial neural network (ANN) [18], decision tree [9, 12], and bayesian classifier [6, 13].

A set of well-designed hand-crafted features is necessary and important for high performance and robustness in traditional methods, while it costs a lot of labor to design manual features. How to design features usually depends on the researchers' work experience. As a consequence, methods based on the deep neural network [19] have gradually become mainstream in ECG classification due to the ability to extract features automatically. Convolutional neural networks (CNNs) are widely employed because of their ability to extract features effectively. A patient-specific ECG heartbeat classification using an adaptive CNN was developed by Kiranyaz et al. [20], which is a single structure that integrates feature extraction and classification. The continuous wavelet transform was utilized by Al Rahhal et al. [21] to convert ECG into images, which were then input into a CNN network pretrained on ImageNet. For identifying supraventricular and ventricular ectopic beats, this approach performed well. A 34-layer residual CNN presented by Hannun et al. [22] reached expert-level performance in detecting cardiac arrhythmias. In some studies, the ECG signal was regarded as a time-series and they deployed recurrent neural network (RNN) which is designed for dealing with sequential data. Long short-term memory (LSTM) and gated recurrent unit (GRU) are two representative variants of RNN. Based on several LSTMs and wavelet transform, a real-time heartbeat classification method was developed by Saadatnejad et al. [23] for personal wearable gadgets. For classifying biometric ECG signals, a deep bidirectional GRU network was developed by Lynn et al. [24]. Besides all that, many studies have proposed multilayer networks by combining CNN and RNN. By combining a residual CNN with a bidirectional LSTM, He et al. [25] achieved good results for arrhythmia classification. Yao et al. [26] used a model composed of VGGNet and LSTMs to classify multiclass arrhythmias. This model is effective in recognizing paroxysmal arrhythmias and supports varied-length inputs. Recently, a number of works [27, 28] have exploited the attention mechanism to take into account the fact that different parts of ECG signals contribute dissimilarly to the diagnosis. There are many variants of the attentional mechanism [29–31]. Zhang et al. [32] used the spatio-temporal attention mechanism to deal with the ECG classification by assigning weights in the spatio-temporal dimension of ECG. These works exploited the attention mechanism to assign weights to ECG signals at the level of time point (i.e., temporal attention mechanism). The temporal attention mechanism can focus on which signal points are more important in the temporal dimension and which signal points do not have a sufficiently prominent contribution to the result. However, the ECG signal is composed of heartbeats; so another practicable alternative is to exploit the attention mechanism to assign weights at the level of ECG heartbeat. Considering the use of the attention mechanism from the perspective of the heartbeat allows the attention mechanism to take the heartbeat as a whole and pay attention to how much the heartbeat contributes to the result. That is to say, beats that contribute more to the result are assigned higher weights. This provides a new perspective to treat and process ECG signals. In other words, extracting features from each beat and fusing these features deserves further research.

## 3. Method

### 3.1. Problem Formulation

The multiclass and multilabel 12-lead ECG dataset is defined as

(1) $$\begin{array}{c} X=\left\{\left(x^{\left(1\right)},y^{\left(1\right)}\right),\left(x^{\left(2\right)},y^{\left(2\right)}\right),\ldots ,\left(x^{\left(n\right)},y^{\left(n\right)}\right)\right\}\text{,} \end{array}$$

where *x*^(*i*)^ ∈ *ℝ*^*L*×*D*^ is the ECG signal, *L* refers to the length of the signal, and *D* refers to the signal dimension (i.e., the number of leads). *y*^(*i*)^ ∈ *𝔽*_2_^*C*^, *C* refers to the number of categories and *𝔽*_2_={0,1} is a set containing only 0 and 1.

The goal of the arrhythmia classification is to construct a model to automatically identify the categories of arrhythmia based on the ECG signal. The model takes 12-lead ECG signals as input and outputs predicted labels. The model needs to learn the mapping relationship *ℋ*(·) from the input *x*^(*i*)^ to the output *z*^(*i*)^ of the output layer, which is defined as

(2) $$\begin{array}{c} z^{\left(i\right)}=H\left(x^{\left(i\right)};\theta \right)\text{,} \end{array}$$

where *θ* refers to the network parameters of the model. During training, the goal of the model is to minimize the binary cross entropy loss (BCE Loss) of the predicted probability relative to its reference label, defined as

(3) $$\begin{array}{c} L\left(X;H\right)=-\overset{C}{\underset{k=1}{\sum }}\left(y_{k}^{\left(i\right)}\log z_{k}^{\left(i\right)}+\left(1-y_{k}^{\left(i\right)}\right)\log\;\left(1-z_{k}^{\left(i\right)}\right)\right)\text{.} \end{array}$$

### 3.2. Model Overview

The proposed BLF-Net includes 3 parts illustrated in Figure 1: (1) segmentation used for segmenting ECG signal into heartbeats; (2) beat-level feature extraction used for extracting features from beats; (3) interbeat feature fusion used for synthesizing features extracted by beat-level feature extraction module.

Specifically, in our model, the ECG signal is first fed into the segmentation module, and several segmented beats are obtained. The segmented beats are sent to the beat-level feature extraction module to obtain the encoded features of each beat. These features are then fed into the interbeat feature fusion module, where the features are fused using an attention mechanism to assign different weights to emphasize useful beats and suppress the less useful ones. Finally, a two-layer fully connected layer is used as a classifier to output the probability of classification.

The ECG signal is a periodic and multibeat signal. The heartbeat is the basic component of the ECG signal. A typical ECG signal consists of a P wave, QRS complex, and other waves. Different heartbeats are temporally and physiologically correlated with each other. On the one hand, the heartbeat can be divided into P, QRS, T waves, etc., according to the physiological process of the heart, which corresponds to the occurrence of different changes in the heart and is expressed as a complete cycle; on the other hand, when pathological changes occur, there may be irregular changes between different beats of one ECG signal. Such changes are expressed as the variability between different beats. According to the above-given two points, pathological changes in the heart can be reflected by the individual beat characteristics of the ECG signal. Therefore, each heartbeat should be emphasized, and the method used for automatic arrhythmia detection should have the ability to extract features from individual heartbeats.

### 3.3. Segmentation

Let *X* ∈ *ℝ*^*L*×*D*^ be an original ECG signal, where *L* is the length of the original ECG signal and *D* is the number of leads. Then, we adopt a classical R-peak detection algorithm proposed by Pan et al. [33]. This algorithm comprises the following steps: (1) bandpass filter, (2) differentiator, (3) squaring process, (4) moving-window integration, and (5) thresholding. After this, we get a sequence of R-peaks.

According to the positions of the detected R-peaks, we segment the original ECG signal into heartbeats. The first *L*_*f*_ points and the last *L*_*k*_ points of an R-peak are considered as one heartbeat. Finally, we have a series of beats denoted as *B*=(*b*_1_, *b*_2_,…, *b*_*s*_) where *b*_*i*_ ∈ *ℝ*^*L*_*b*_×*D*^, *i* ∈ 1,2,…, *s*, *L*_*b*_=*L*_*f*_+*L*_*k*_ is the length of a heartbeat.

### 3.4. Beat-Level Feature Extraction

Beat-level feature extraction module is composed of CNN and RNN. Hence, the procedure for this part can be formulated as

(4) $$\begin{array}{c} f_{CNN}=CNN\left(B\right)=CNN\left(b_{1},b_{2},\ldots ,b_{s}\right)\\ =\left(CNN\left(b_{1}\right),CNN\left(b_{2}\right),\ldots ,CNN\left(b_{s}\right)\right)\\ =\left(f_{CNN_{1}},f_{CNN_{2}},\ldots ,f_{CNN_{s}}\right),\\ f_{RNN}=RNN\left(f_{CNN}\right)\\ =RNN\left(f_{CNN_{1}},f_{CNN_{2}},\ldots ,f_{CNN_{s}}\right)\\ =\left(RNN\left(f_{CNN_{1}}\right),\ldots ,RNN\left(f_{CNN_{s}}\right)\right)\\ =\left(f_{1},f_{2},\ldots ,f_{s}\right). \end{array}$$

#### 3.4.1. Convolutional Neural Network

A convolutional neural network contains 6 1-dimension (1-D) convolution layers, as shown in Figure 1. “Conv1d 3 × 64, 2” means that the kernel size of the convolution layer is 3, the number of kernels is 64, and the stride for the cross-correlation is 2. “Conv1d 3 × 64” means that the stride for the cross-correlation is 1. Other similar expressions have similar meanings. A batch normalization (BN) layer together with a rectified linear unit (ReLU) function follows each convolution layer. BN [34] normalizes each batch during training, which is used for accelerating the convergence. ReLU [35] is a common function used for activating output values and avoiding the vanishing gradient to a certain extent. Dropout [36] follows every two convolution layers to prevent overfitting.

#### 3.4.2. Recurrent Neural Network

Following the convolutional neural network, the recurrent neural network (RNN) is utilized. More specifically, GRU [37], a kind of RNN, is adopted here. GRU uses gate mechanisms to modulate the information flow, similar to LSTM, but the hidden state is utilized to convey information instead of the cell state. We use a bidirectional GRU which is a combination of a forward GRU layer and a backward GRU layer.

(5a) $$\begin{array}{c} y_{t}=f\left(W_{z}x_{t}+U_{z}⊙h_{t-1}\right)\text{,} \end{array}$$

(5b) $$\begin{array}{c} r_{t}=f\left(W_{r}x_{t}+U_{r}h_{t-1}\right)\text{,} \end{array}$$

(5c) $$\begin{array}{c} {\tilde{h}}_{t}=\tanh\;\left(Wx_{t}+U\left(r_{t}h_{t-1}\right)\right)\text{,} \end{array}$$

(5d) $$\begin{array}{c} h_{t}=\left(1-y_{t}\right)h_{t-1}+y_{t}{\tilde{h}}_{t}\text{.} \end{array}$$

Here, the sigmoid function is denoted by the symbol *f*. ⊙ stands for element-by-element multiplication. The update and reset gates, *y*_*t*_ and *r*_*t*_, determine the extent to which the activation *h*_*t*_ is updated and the extent to which the prior activation *h*_*t*−1_ is forgotten, respectively. *W*_*z*_, *U*_*z*_, *W*, *U*, *W*_*r*_ and *U*_*r*_ are the trainable parameters. The activation *h*_*t*_ is the weighted sum of the prior activation *h*_*t*−1_ and the candidate's activation ${\tilde{h}}_{t}$.

### 3.5. Interbeat Feature Fusion

For learning features from several beats and putting different weights on the features of different beats, we utilize the attention mechanism [38] to fuse features extracted from different beats. Considering that the number of heartbeats may not be consistent for each segmented record, the masking technique is used. After using the masking technique, the attention mechanism actually performs assigning weights to the heartbeats that the record actually has. First, we concatenate the features extracted previously. Let *f*_1_, *f*_2_,…, *f*_*s*_ refer to features. Here, *f*_*i*_ ∈ *ℝ*^*n*^, *n* is the number of features after passing through the beat-level feature extraction module. After passing the concatenation layer, we obtain the following output:

(6) $$\begin{array}{c} f_{o}=Cat\left(f_{1},f_{2},\ldots ,f_{s}\right)\text{.} \end{array}$$

Then, the concatenated features *f*_*o*_ is fed through an attention layer i.e.,

(7) $$\begin{array}{c} f_{att}=Attention\left(f_{o}\right)\text{.} \end{array}$$

This algorithm is formulated as

(8a) $$\begin{array}{c} u_{i}=\tanh\;\left(Wf_{i}+b\right)\text{,} \end{array}$$

(8b) $$\begin{array}{c} \alpha_{i}=\frac{\exp\;\left(u_{i}^{T}u\right)}{\underset{i}{\sum }\exp\;\left(u_{i}^{T}u\right)}\text{,} \end{array}$$

(8c) $$\begin{array}{c} f_{att}=\underset{i}{\sum }\alpha_{i}f_{i}\text{.} \end{array}$$

Here, *i* ∈ 1,2,…, *s*. This procedure is illustrated in Figure 1. Weights are assigned to beats in an ECG signal by the attention mechanism in order to emphasize those that are more related to arrhythmia detection. In the attention mechanism, we first compute scores using the input of attention layer *f*_*i*_. Specifically, *W* and *b* here are trainable parameters. We compute the linear mapping of *f*_*i*_ and then it is activated by nonlinear function tanh(·). tanh shown in Figure 1 represents this process. In order to get the weight in the interval [0, 1], the softmax function is applied to the scores we get previously. softmax shown in Figure 1 represents this step. Finally, the output of the attention layer is obtained by using different weight factors in the input features *f*_*i*_ to achieve the weighted average. The intersection of the dashed line and the solid line represents a multiplication of scalars and vectors, and the plus sign in the circle means the addition of a vector.

## 4. Experimental Studies and Results

### 4.1. Environment

Python 3.7 and Pytorch 1.2.0 are used to implement the proposed approach. In this study, all of the experiments were carried out on a server using 128 GB of RAM, a Xeon E5 2620 processor, and four GeForce RTX 2080 graphics cards.

### 4.2. Data Description

The PTB-XL dataset [39] consists of 21837 clinical 12-lead ECG records from 18885 patients, each lasting 10 seconds. The annotation of ECG statements follows the SCP-ECG standard [40], and each record can have several statements. The ECG statements in the dataset are divided into 71 different classes. There are 44 diagnostic statements, 19 form statements, and 12 rhythm statements in these categories. The statements are nonexclusive at three levels, and the diagnostic statements comprise four form rhythm statements. Furthermore, diagnostic statements are divided into five superclasses (CD: conduction disturbance, HYP: hypertrophy, MI: myocardial infarction, NORM: normal ECG, and STTC: ST/T change) and 23 subclasses. The number of ECG records and the descriptions of different classes for superclasses of diagnostic statements are shown in Table 1. This study employed a sampling rate of 100 Hz.

### 4.3. Evaluation Metric

We use area under curve (AUC) to evaluate how our model performs on arrhythmia classification. AUC refers to the area under a receiver operating characteristic curve [41]. Let *n* be the number of samples, *M* refers to the number of positive samples, and *N* refers to the number of negative samples; here, *n*=*M*+*N*. First, the samples are sorted in descending order by score. Then, the rank corresponding to the sample with the largest score is set as *n*, and the rank corresponding to the sample with the second-largest score is set as *n* − 1, and so on. Then, we add up the ranks of all the positive samples, subtract *M*(1+*M*)/2, and then divide by *M* × *N*. To sum up, AUC is defined as

(9) $$\begin{array}{c} AUC=\frac{\sum_{i\in positiveClass}\mathrm{ran}k_{i}-M\left(1+M\right)/2}{M\times N}\text{.} \end{array}$$

The Mann–Whitney U, which determines whether negatives are rated lower than positives, is found to be closely related to the AUC. The Wilcoxon test of ranks [42] is another name for it.

### 4.4. Training Setting

#### 4.4.1. Model Optimization

Mini-batch is used for saving memory and accelerating training. The batch size is set to 256 samples. The Xavier uniform initializer [43] is used to initialize the weights of convolutional layers, while the orthogonal initializer is used to initialize the weights of the bidirectional GRU. We also employ the Adam optimizer [44] to iteratively update the parameters due to its potential to speed up the convergence of the network. The rate of learning is set at 3e-4.

#### 4.4.2. Regularization Strategies

Because the neural network has huge amounts of parameters, to avoid overfitting, we need to apply regularization on the loss function to impose a cost on the optimization function to make the optimal solution smooth. Specifically, *L*_2_ regularization is utilized in our model. *L*_2_ regularization is the most common regularization technique. *L*_2_ regularization limits the magnitude of the parameters by adding a penalty term to the loss function. With *w* representing the parameters of the model, *L*_2_ regularization is expressed as

(10) $$\begin{array}{c} L_{2}\left(\theta \right)={\left\|\theta \right\|}_{2}^{2}=\underset{i}{\sum }\theta_{i}^{2}\text{.} \end{array}$$

The loss function with *L*_2_ regularization term is expressed as

(11) $$\begin{array}{c} L_{R}\left(X;H\right)=L\left(X;H\right)+L_{2}\left(\theta \right)\text{.} \end{array}$$

Here, *L*_*R*_(*X*; *ℋ*) is the loss function used in our model, *L*(*X*; *ℋ*) is the BCE loss as noted in equation (3).

#### 4.4.3. Cross Validation

The PTB-XL dataset was divided into ten parts by reference [39]. The tenth part serves as the test set and the rest of the nine parts serve as the training set. For the remaining nine parts, we follow the recommendation and use 9-fold cross-validation to make use of the training set thoroughly in consideration of the small size of the training set. We divide the training set into nine equal parts using this strategy. Each of the nine parts takes turns as the validation data, and the training data is made up of the remaining subsets. In the end, the final probabilities are calculated by averaging the output of nine models.

### 4.5. Experimental Process

The input shape of the network is (256, 12, 1000). The first dimension is the batch size for the mini-batch, here is 256. The second dimension refers to the channel number (i.e., the number of leads). The third dimension here is the length of the signal whose sampling frequency is 100 Hz and duration is 10 s.

After passing the segmentation module, the dimensions are turned into (256, 20, 12, and 80). Here, the first dimension is still the batch size and the third dimension is the channel number. The second dimension is the number of beats and the fourth dimension is the length of beat, which is set to 25 before R-peak and 55 after R-peak. Then, these segmented ECG signals are fed into the beat-level feature extraction module. Since one out of every two convolutional layers is set to stride 2, the output of the convolutional block is with dimensions (256, 20, 256, and 10). The first and the second dimensions are the same as before and the third dimension is the kernel number of the last layer. These feature maps are flowed into a GRU and a linear layer to get features with dimensions (256, 20, 64, and 10).

Next, these features are put into the interbeat feature fusion module to fuse features extracted from the beat-level feature extraction module along the dimension of different beats. The input of the beat-level feature fusion module is reshaped into (256, 20, 640). That is, we merge the last two dimensions as features of a certain beat. All these features are fed into the attention layer to obtain the fusion features with dimensions (256, 640). Finally, a fully connected layer is adopted as a classifier to transform these features into probabilities of different kinds of arrhythmias. Here, the sigmoid function is utilized to compress the output of the model into probabilities between 0 and 1. Adam optimizer is adopted to iteratively update network parameters.

## 5. Result & Discussion

### 5.1. Classification Performance

With the above-given experimental setup, the experiments were conducted. We followed the recommendations of [45] and compared them with 7 previous works at 6 annotation levels.  Table 2 compares the proposed method with 7 previous works [45] on six classification tasks based on macro-AUC scores. As shown in Table 2, our algorithm has superiority over the works listed in [45]. Compared to the wavelet + NN algorithm, macro-AUC scores are improved by 9.2%, 9.7%, 9.5%, 7.1%, 17.7%, and 8.9% in the six classification tasks, respectively. The number of parameters in our model is better than that of methods with similar performance, as will be discussed later. This demonstrates that the proposed algorithm produces a significant improvement in detecting most arrhythmias, suggesting that it is a competitive method in detecting arrhythmias when compared to state-of-the-art methods. And, the confusion matrices are shown in Figure 2.

### 5.2. Ablation Studies

To explain the effectiveness of BLF-Net and investigate the influence of hyperparameters in model performance, ablation studies are applied. In this process, we deploy the same experimental settings as before. That is, the same evaluation metric and training settings are adopted.

#### 5.2.1. Comparison between Backbone Network and BLF-Net

To illustrate the validity of BLF-Net, we make experiments to compare the performance between the backbone network and BLF-Net. The backbone network is the same structure as the beat-level feature extraction module shown in Figure 1, which is followed by a fully connected layer as a classifier. There is no beat-level fusion structure in the backbone network. That is, we send the original ECG signal to the backbone network without segmentation and interbeat feature fusion. By contrast, we deploy the model with segmentation and feature fusion i.e., BLF-Net.  Table 3 shows the macro-AUC score of the backbone network and BLF-Net in classifying multi-class cardiac arrhythmias based on the PTB-XL dataset.

This experiment demonstrates the introduction of the beat-level fusion module can effectively improve the accuracy of arrhythmia detection by contrast with a simple feature extraction module. As shown in Table 3, BLF-Net outperforms BackboneNet based on the macro-AUC score of all different criteria in detecting multiclass cardiac arrhythmias.

#### 5.2.2. Comparison between Temporal Attention Module and with Interbeat Feature Fusion Module

To verify the effectiveness of the interbeat feature fusion module, we make another experiment to compare the performance between the temporal attention module and the interbeat feature fusion module. In this experiment, we remove the segmentation module of BLF-Net and feed the original ECG signal into the neural network. Then, the interbeat feature fusion module is changed to the temporal attention module. The modified model is named temporal attention network, and we compare the results of this model with BLF-Net. The structure of the temporal attention network consists of the backbone network and the temporal attention module. The backbone network is the same configuration as the BLF-Net, which is followed by the temporal attention module used for assigning weights to the features temporally. A fully connected classifier is employed here and the number of output categories is denoted as *n*_*c*_. The result is shown in Table 4. This experiment is conducted to demonstrate that the attention module applied among beats outperforms that applied among time points. The temporal attention module assigns weights temporally. This means that the attention module focuses on the microlevel, which is less likely to capture global information and focuses more on local changes. While the interbeat feature fusion module focuses on the beat level, this allows for a better fusion of features extracted from each beat.

#### 5.2.3. Analysis of Segmentation Length

The heartbeat length *L*_*b*_ in this experiment is set to 80 points. This hyperparameter can be regarded as a window size for a beat-level feature extraction module to observe heartbeats. Here, experiments were conducted to analyse the effect of this hyperparameter on the model. We chose different heartbeat length *L*_*b*_ to repeat the experiments of arrhythmias detection based on the PTB-XL dataset.  Table 5 shows the result of these experiments. It can be seen that among the rhythm *L*_*b*_=160 reachs the highest score and among the form *L*_*b*_=80 reaches the highest score. From here, we can get a conclusion, the greater the heartbeat length we set, the better score among the rhythm we get. And, the smaller heartbeat length we set, the better score among the form we get. we can infer that a greater heartbeat length will catch more information about rhythm and a smaller heartbeat length will catch less.

An explanation is given for the decrease in macro-AUC scores as the heartbeat length is reduced. A shorter heartbeat length means a smaller observation window for the ECG signal. The signal acquired by a single heartbeat becomes less. Unlike morphological judgments, rhythm is inferred by comparing similar signals at the time before and after. While morphology is judged by the amplitude at the same time. For shorter time windows, we have less signal to observe and less signal to compare back and forth. For longer time windows, more signals can be observed and more signals can be compared back and forth to determine rhythm-related information, so the larger the observation window, the more accurate the rhythm-related judgments. Longer signals mean that it is easier to determine the rhythm of the heartbeat.

### 5.3. Performance Analysis

ECG signal is composed of beats, each heartbeat reflects the same electrical activity (i.e., from depolarization to repolarization). One cycle of the electrical activity of the heart can be denoted as a random signal *X*(*t*). Beat in the sample can be regarded as the observed signal *x*(*t*) of random signal *X*(*t*). Beats that come from the same ECG signal have the same physiological meanings and individuals, so they can be considered as an identical distribution. Therefore, a series of continuous beats can be dealt with the same network due to identical distribution. In this paper, a module named beat-level feature extraction is deployed to extract features from beats. Our beat-level feature extraction module extract features from beats with the same structure. Then, features extracted by the beat-level feature extraction module are fed into the interbeat feature fusion module to focus more on the representative beats. Take the STTC as an example. The ST segment myocardial infarction (STEMI) is reflected in ST elevation [46]. ST elevation is linked to infarction and can be preceded by changes indicating ischemia, such as ST depression or the T waves inversion, according to [47]. In this case, our model will assign higher weights to those heartbeats that show the morphological characteristic of ST elevation.

### 5.4. Attention Weights

To illustrate how the interbeat feature fusion module works, we show the weights assigned by the attention layer, as shown in Figure 3. The upper parts in Figures 3(a)–3(d) show the waveform of lead II, and the lower parts show the weights assigned by our interbeat feature fusion module. The higher weight assigned to a beat, the more contribution this beat has to the result. As shown in Figure 3, our model gives higher weights to the abnormal heartbeats, suggesting that these abnormal heartbeats are paid more attention to in our method. In clinical practice, abnormal heartbeats define the diagnostic results for the ECG signal. Therefore, we can consider that the proposed method well learns the important features from ECG signals and reasonably explains the classification results.

### 5.5. Parameter Size

We make a comparison in terms of the number of parameters between the proposed BLF-Net and four previous works in this subsection, as shown in Table 6. It can be seen that the proposed model does not have a large number of parameters but achieves optimal performance. Compared to “inception1d” and “resnet1d_wang,” our model outperforms on the macro-AUC score. And, as shown in Table 2, our model surpasses the performance of other models on subdiagnostic and superdiagnostic significantly. Although the performance of the model “xresnet1d101” is comparable to ours, the number of parameters in our model is much less than this works. The experiment result shows that a decrease in convolutional layers doesn't sacrifice the ability of models to learn compared with other models. In addition, fewer parameters are less likely to overfit, contributing to better generalization and less memory-consuming.

## 6. Conclusion

BLF-Net, an end-to-end multiclass arrhythmia classification model utilizing 12-lead ECG records, is proposed in this study. The attention mechanism is used by BLF-Net to focus on the informative features while suppressing the unimportant ones. Experiments show that when compared to off-the-shelf methods, BLF-Net achieves state-of-the-art performance. And, BLF-Net is both lightweight and effective. BLF-Net, the proposed model for arrhythmia classification, has the promise of aiding cardiologists in their clinical practice.

## Figures and Tables

**Figure 1:** The framework of our method.

**Figure 2:** The confusion matrices of BLF-net on superdiagnostic. The first subfigure shows an example of a subfigure. TN, FP, FN, and TP represent true negative, false positive, false negative and true positive, respectively.

**Figure 3:** The heartbeat-level weights assigned by the proposed interbeat feature fusion module for different ECG classes including (a) myocardial Infarction, (b) conduction disturbance and myocardial infarction, (c) myocardial infarction and ST/T change, and (d) conduction disturbance and hypertrophy and myocardial Infarction. The upper subfigures in (a)–(d) show the original ECG signal from lead II. The lower subfigures show the corresponding heartbeat-level weights.

**Table 1:** List of the distribution and the description for superclasses of diagnostic statements.

#Records	Superclass	Description
9528	NORM	Normal ECG
5486	MI	Myocardial infarction
5250	STTC	ST/T change
4907	CD	Conduction disturbance
2655	HYP	Hypertrophy

**Table 2:** Comparing our work with the previous works in terms of classification performance.

Models	Macro-AUC scores					
	All	Diag.	Sub-diag.	Super-diag.	Form	Rhythm
Lstm^1^	0.907	0.927	0.928	0.927	0.851	0.953
Inception1d^1^	0.925	0.931	0.930	0.921	**0.899**	0.953
Lstm_bidir^1^	0.914	0.932	0.923	0.921	0.876	0.949
Resnet1d_wang^1^	0.919	0.936	0.928	0.930	0.880	0.946
Fcn_wang^1^	0.918	0.926	0.927	0.925	0.869	0.931
Wavelet + NN^1^	0.849	0.855	0.859	0.874	0.757	0.890
Xresnet1d101^1^	0.925	0.937	0.929	0.928	0.896	0.957
Ours	**0.927**	**0.938**	**0.941**	**0.936**	0.891	**0.969**

^1^These models are stated in detail in [45]. The best performance is highlighted in bold.

**Table 3:** Comparing our work with the branch network in terms of classification performance.

Models	Macro-AUC scores					
	All	Diag.	Sub-diag.	Super-diag.	Form	Rhythm
BackboneNet	0.908	0.924	0.921	0.919	0.828	0.946
BLF-net	**0.927**	**0.938**	**0.941**	**0.936**	**0.891**	**0.969**

The best performance is highlighted in bold.

**Table 4:** Comparing our work with the temporal attention network in terms of classification performance.

Models	Macro-AUC scores					
	All	Diag.	Sub-diag.	Super-diag.	Form	Rhythm
Temporal attention network	0.921	0.920	0.923	0.930	0.855	0.953
BLF-net	**0.927**	**0.938**	**0.941**	**0.936**	**0.891**	**0.969**

**Table 5:** Comparison of BLF-Net with different heartbeat lengths in terms of classification performance.

Lengths	Macro-AUC scores					
	All	Diag.	Sub-diag.	Super-diag.	Form	Rhythm
*L*_*b*_=160	0.925	0.937	0.931	0.933	0.887	**0.969**
*L*_*b*_=120	0.923	**0.938**	0.934	0.931	0.890	0.961
*L*_*b*_=80	**0.927**	0.937	**0.941**	**0.936**	**0.891**	0.954

The best performance is highlighted in bold.

**Table 6:** Comparison of the number of parameters of previous works and the proposed BLF-Net.

Models	The number of parameters
Inception1d^1^	507653
Resnet1d_wang^1^	473349
Fcn_wang^1^	309765
Xresnet1d101^1^	3642501
Ours	569373

^1^These models are stated in detail in [45].

## Data Availability

The PTB-XL database used to support the findings of this study is publicly available and can be downloaded at https://physionet.org/files/ptb-xl/1.0.1/.
